# A New Approach for the Discovery of Antibiotics by Targeting Non-Multiplying Bacteria: A Novel Topical Antibiotic for *Staphylococcal* Infections

**DOI:** 10.1371/journal.pone.0011818

**Published:** 2010-07-27

**Authors:** Yanmin Hu, Alireza Shamaei-Tousi, Yingjun Liu, Anthony Coates

**Affiliations:** 1 Medical Microbiology, Centre for Infection, Division of Cellular and Molecular Medicine, St George's, University of London, London, United Kingdom; 2 Helperby Therapeutics Group plc, London, United Kingdom; University of Hyderabad, India

## Abstract

In a clinical infection, multiplying and non-multiplying bacteria co-exist. Antibiotics kill multiplying bacteria, but they are very inefficient at killing non-multipliers which leads to slow or partial death of the total target population of microbes in an infected tissue. This prolongs the duration of therapy, increases the emergence of resistance and so contributes to the short life span of antibiotics after they reach the market. Targeting non-multiplying bacteria from the onset of an antibiotic development program is a new concept. This paper describes the proof of principle for this concept, which has resulted in the development of the first antibiotic using this approach. The antibiotic, called HT61, is a small quinolone-derived compound with a molecular mass of about 400 Daltons, and is active against non-multiplying bacteria, including methicillin sensitive and resistant, as well as Panton-Valentine leukocidin-carrying *Staphylococcus aureus*. It also kills mupirocin resistant MRSA. The mechanism of action of the drug is depolarisation of the cell membrane and destruction of the cell wall. The speed of kill is within two hours. In comparison to the conventional antibiotics, HT61 kills non-multiplying cells more effectively, 6 logs versus less than one log for major marketed antibiotics. HT61 kills methicillin sensitive and resistant *S. aureus* in the murine skin bacterial colonization and infection models. No resistant phenotype was produced during 50 serial cultures over a one year period. The antibiotic caused no adverse affects after application to the skin of minipigs. Targeting non-multiplying bacteria using this method should be able to yield many new classes of antibiotic. These antibiotics may be able to reduce the rate of emergence of resistance, shorten the duration of therapy, and reduce relapse rates.

## Introduction 

The traditional route for identifying early hits in antibiotic research is to target multiplying bacteria. All current antibiotics have been generated this way. Activity of a potential antibiotic in such assays is predictive of an antimicrobial effect in humans (bearing in mind many compounds are not suitable due to undesirable characteristics such as toxicity). The disadvantage of this route is that the numbers of novel classes of non-toxic compounds which kill multiplying bacteria may have been almost exhausted [1] and those that remain, may require substantial effort and expense to bring to market. Furthermore anti-multiplying agents are almost always either inactive or only partially active against non-multiplying or slowly multiplying or persister bacteria [2], [3], [4], [5], [6] which leads to the need for multiple doses of antibiotics in order to achieve cure of a bacterial infectious disease. This prolongs the duration of therapy and increases the emergence of resistance. Since bacterial resistance reduces the effectiveness of antibiotics, new ones are required at regular intervals, as the old ones lose their potency for most infections. However, the number of new antibiotics which reach the market each year is falling [1], [3], [5], [7], [8]. Whilst at least 15 classes of antibiotics were introduced into the market between 1940 and 1962 [3], only three new classes of antibiotics have been marketed since then [9], [10], [11]. Together with their subsequent analogues, each class loses effectiveness, at least for some species of bacteria such as Gram-negatives, within 50 years after entry into the market. So, if we continue to use existing technologies for the next 50 years, it is unlikely that we will produce enough new classes to prevent the antibiotic era fading away. A fundamentally new route for antibiotic drug discovery is required if the antibiotic era is to continue. Bacterial molecules have been targeted, in order to create new drugs, but this has not produced any new classes of antibiotics which have reached the market [7]. Another potential way to develop new antibacterials is to use bacteriophages. Although this method has been utilized for decades, no marketed bacteriophages are available in Western countries for licensed medicinal purposes.

We have proposed a new approach for the production of novel classes of antibiotics [1], [3]. This new route targets whole bacteria which are in the non-multiplying stage from the beginning of the discovery process. In a clinical infection, there is co-existence of multiplying bacteria and non-multiplying bacteria [5], [12]. Although non-multipliers do not cause overt disease, they act as a pool from which multiplying bacteria emerge to cause recurrent disease. Current antibiotics kill multiplying bacteria, but they are very inefficient at killing non-multipliers [3], [4], [13], [14] which leads to slow or partial death of the total target population in an infected tissue. This results in repeated administration of antibiotics and leads to extended periods of antibiotic treatment. For example, tuberculosis has a drug regimen lasting at least six months [15]. Bacterial endocarditis is treated for several weeks. Non-multipliers probably also occur in many other common infections such as sore throat and infected eczema [3], [5], [7], [16]. In turn, these repeat-dose drug treatments can result in the emergence of antibiotic resistance associated with poor patient compliance [3], [16]. These contribute to the short life span of antibiotics when they reach the market. An ideal antibiotic would swiftly kill all of the non-multiplying and multiplying bacteria in an infected tissue, thereby shortening antibiotic regimens. This process should slow the emergence of genetic resistance, because mutation cannot occur if there are no live target bacteria. Unfortunately, no marketed antibiotic lives up to this ideal, and resistance is now widespread.

Here we describe a proof of principle study for a new approach in which we have selected for a compound throughout the discovery process that has activity against non-multiplying bacteria. The lead compound, HT61 which is a topical antibiotic, is more bactericidal for non-multiplying bacteria than marketed antibiotics but is less potent against multiplying organisms. It does not induce resistance over 50 passages of suboptimal treatment. HT61 kills non-multiplying bacteria in an animal model, and is not toxic when applied to the skin of minipigs. This compound is now in clinical trials.

## Results

### Establishment of a long term non-multiplying stationary phase model for drug selection

In order to establish stationary phase models, methicillin-sensitive *Staphylococcus aureus* (MSSA) and methicillin-resistant *S. aureus* (MRSA) were grown in nutrient broth for 10 days. Viability of the bacteria was determined by CFU counts at different time points. As shown in Fig 1, the growth in both aerated cultures reached peaks (1.5×10^9^ CFU/ml) at 24 hours of growth, the CFU counts remained relatively constant until 6 days of incubation for MSSA and 7 days for MRSA, then gradually decreased to a value of about 3×10^8^ CFU/ml after 10 days of incubation.

**Figure 1:** Growth curves of methicillin-sensitive and methicillin-resistant *S. aureus*. The bacterium was grown in nutrient broth medium with shaking for 10 days. The arrows indicate the timepoints when the cultures were used for drug sensitivity test. These results were confirmed in two independent experiments.

Long-term stationary phase cultures of 5 to 6 days were chosen. These late stationary phase cultures, as seen in Fig. 1, may represent a mixed population with a dynamic balance of cell division and cell death [17]. In order to induce the bacterial cells into a non-replicating stage, we washed and incubated the cells with PBS. No changes in CFU counts of the bacteria were observed after 24 hours of incubation in the buffer (data not shown) indicating that the bacteria were in a non-multiplying state. The nutrient depleted 5–6 day stationary phase cell suspension was used to screen or test drugs and was called non-multiplying stationary phase bacteria.

### Strategy of screening drugs against non-multiplying bacteria

A previous study has demonstrated that fluoroquinolones such as ciprofloxacin, ofloxacin, levofloxacin, moxifloxacin, and gatifloxacin exhibit bactericidal activity against stationary phase and persistent *Mycobacterium tuberculosis* [18]. We used a company, Argenta Discovery UK, to search similar commercially available structures to quinolones using a virtual screening technique. All 2-D substructure and similarity searches were carried out in the Argenta “Unity” database which comprised 952,601 commercially available, drug-like compounds collated from the collection of over 40 suppliers worldwide. As a result of the computer aided search, we chose 57 quinolone-like compounds which we obtained commercially. We screened activities of these compounds against non-multiplying MSSA using the model described above. We found that only two of these compounds with similar structures showed stationary phase bactericidal effects with 2–3 log kill of non-multiplying bacteria. We used these active compounds as core structures to synthesise analogues. Over 300 new derivative compounds were synthesised by Argenta Discovery UK and were screened for activity against non-multiplying *S. aureus*. We have seleted many compounds showing bactericidal activity. One of them, named HT61, is a quinolone-derived compound which presented significant potency.

### HT61 is more active against non-multiplying MSSA and MRSA than selected marketed antibiotics

The activity of HT61 against non-multiplying MSSA was compared with several marketed antibiotics. Non-multiplying MSSA was incubated with different concentrations of HT61, amoxicillin/clavulanic acid (Augmentin), azithromyicin, levofloxacin, linezolid, daptomycin and mupirocin for 24 hours, and the activities of the drugs were measured by CFU counts. As shown in Fig. 2A, HT61 kills over 7 log CFU/ml at a concentration of 12.5 µg/ml. The minimum stationary phase-cidal concentration 50 (MSC_50_) of HT61 is 2.5 µg/ml and the minimum stationary phase-cidal concentration 99 (MSC_99_) was 4.5 µg/ml. In contrast, amoxicillin/clavulanic acid (Augmentin), azithromyicin, levofloxacin, linezolid and mupirocin at 50 µg/ml failed to exhibit any activities against the non-multiplying bacteria. Daptomycin reduced the CFU counts from log 7 to 0 at 50 µg/ml. The minimum stationary phase-cidal concentration 50 (MSC_50_) of daptomycin is 2.5 µg/ml and the minimum stationary phase-cidal concentration 99 (MSC_99_) was 9 µg/ml.

**Figure 2:** Effects of HT61 and marketed antibiotics against stationary phase non-multiplying MSSA and MRSA. HT61 and the antibiotics were added to the non-multiplying cultures at different concentrations. CFU counts were carried out after 24 hours of incubation. A. Effects of HT61, amoxicillin/clavulanic acid, azithromyicin, levofloxacin, linezolid, daptomycin and mupirocin against MSSA. B. Effects of HT61, vancomycin, daptomycin and mupirocin against MRSA. These results were confirmed in two independent experiments.

We also tested the activities of HT61, vancomycin, daptomycin and mupirocin against non-multiplying MRSA. As shown in Fig. 2B, HT61 at 12.5 µg/ml reduced the CFU counts of MRSA from log 7 to 0. The MSC_50_ of HT61 against MRSA was 2.6 µg/ml and the MSC_99_ was 6 µg/ml. However, both vancomycin and mupirocin at 100 µg/ml showed no activity against the same cultures. Daptomycin killed the MRSA at 50 µg/ml showing a MSC_50_ at 2.5 µg/ml and a MSC_99_ at 9 µg/ml. The data indicate that HT61 is more active against non-multiplying MSSA and MRSA than commonly marketed antibiotics.

### HT61 is less potent against multiplying *S. aureus*

The MIC of HT61 and these conventional antibiotics against multiplying *S. aureus* were determined. Log phase *S. aureus* was very sensitive to amoxicillin/clavulanic acid (Augmentin) (MIC 0.8 µg/ml), azithromyicin (MIC 1.56 µg/ml), levofloxacin (MIC 0.2 µg/ml), linezolid (MIC 0.8 µg/ml), daptomycin (1 µg/ml) and mupirocin (MIC 0.2 µg/ml). However, HT61 is less potent against multiplying *S aureus* than marketed antibiotics with an MIC of 8 µg/ml.

### Quick action of HT61 against non-multiplying *S. aureus*

In order to investigate the speed of kill, different concentrations of HT61 were incubated with non-multiplying MSSA for 24 hours. At various time points, the viability of the bacteria was examined by CFU counts. As shown in Fig. 3A, at 10 µg/ml HT61 killed 10^7^ *S. aureus* after 5 hours of treatment and at 20 µg/ml HT61 kill the same numbers of *S. aureus* after one hour of treatment. A similar speed of kill was shown for MRSA (Fig. 3B).

**Figure 3:** Speed of kill with HT61 against non-multiplying MSSA and MRSA. HT61 was incubated with MSSA (A) and MRSA (B) at different concentrations for 24 hours. At different time points, CFU counts were performed.

### HT61 kills non-multiplying clinical MRSA isolates including those which are mupirocin resistant

HT61 was tested against 103 clinical isolates of MRSA which had been isolated from St George's Hospital, London. HT61 was incubated with 10^6^ non-multiplying MRSA for 24 hours, and the drug activity was examined by CFU counts. As shown in Table 1, MSC_50_ of HT61 was 1.5 to 7.5 µg/ml against these 103 MRSA isolates. Amongst these 103 MRSAs, there are 8 strains which were resistant to mupirocin (5 high level and 3 low level resistance). HT61 was active against all of the mupirocin resistant MRSAs.

**Table 1:** The MSC_50_ and MIC of HT61 against clinically isolated MRSA, VISA and VRSA.

MSC_50_ (**µ**g/ml)	Number of MRSA	MIC (**µ**g/ml)	Numbers of MRSA	Numbers of VISA and VRSA
1.5–1.9	26	4	32	9
2–2.9	12	8	13	5
3–3.9	30			
4–4.9	19			
5–5.9	5			
6–6.9	5			
7–7.9	4			

The MIC of HT61 was determined using 45 MRSA, 11 vancomycin-intermediate *S. aureus* (VISA) and 3 vancomycin resistant *S. aureus* (VRSA) which were clinical isolates collected from different hospitals in the UK. As shown in Table 1, the MIC of these MRSA, VISA and VRSA was 4 and 8 µg/ml.

### HT61 was active against other gram positive bacteria

HT61 was incubated with non-multiplying stationary phase *Streptococcus pyogenes*, *Streptococcus agalactiae* and *Propionibacterium acnes* at 20, 10, 5 and 0 µg/ml for 24 hours. As shown in Fig. 4, HT61 at 20 µg/ml reduced the CFU counts of *S. pyogenes* and *S. agalactiae* from log 6 to 0. There were more than one log kills at 10 µg/ml for these strains. HT61 at 10 µg/ml reduced the CFU counts of *S. epidermidis* and *P. acnes* to 0. The MICs of HT61 against these strains were 8 µg/ml.

**Figure 4:** Effects of HT61 against stationary phase non-multiplying *S. pyogenes*, S. *agalactiae*, *S. epidermidis* and *P. acnes*. HT61 was added to the non-multiplying cultures at 20, 10, 5 and 0 µg/ml. CFU counts were carried out after 24 hours of incubation. These results were confirmed in two independent experiments.

### No resistant *S. aureus* was selected after long-term treatment with HT61

The initial MSC_50_ for HT61 was 2.5 µg/ml when inoculated with 10^7^ non-multiplying MSSA. The MIC of this strain for HT61 was 8 µg/ml. Selection of resistance was performed using log phase and stationary phase cultures which were exposed to HT61 at concentrations which were 2 fold below MIC (4 µg/ml) and MSC_50_ (2.5 µg/ml), respectively. After 50 passages of exposure to HT61, no resistance to HT61 was observed in *S. aureus* (data not shown). The same MSC_50_ and MIC was observed at the beginning and at the end of the selection.

### HT61 has no activity against Gram negative bacteria

Bactericidal activity of HT61 was also tested against Gram negative bacteria. The bacterial strains used were *Escherichia coli*, *Klebsiella aerogenes* and *Pseudomonas aeruginosa* which were clinical isolates from St George's Hospital, London. HT61 was incubated with log phase and non-multiplying bacteria at different concentrations from 5 to 40 µg/ml. No activity of HT61 was observed against either log-phase or stationary phase Gram negative bacteria (data not shown).

### Mechanism of action

The affect of HT61 on the cytoplasmic membrane of bacterial cell was investigated. Log phase and 6 day old non-multiplying stationary phase cultures were treated with the fluorescent probe DiSC3(5) which accumulates in bacterial cells and self-quenches its own fluorescence. HT61 at concentrations of 0.156 to 80 µg/ml was added to DiSC3(5) treated cultures. As shown in Fig. 5A, one minute after the addition of HT61, the fluorescence values for the stationary phase cultures increased in a concentration dependent manner, even at levels below the MSC_50_. After one minute of treatment, the fluorescence signal did not increase significantly. These data show that maximum depolarization of the cytoplasmic membrane of stationary phase bacteria occurred within 1 to 4 minutes after treatment with HT61. However, for log-phase cultures (Fig. 5B), the release of fluorescence after treatment of HT61 was slower than that of the stationary phase and reached a peak after 45 minutes. It appears that the increase of fluorescent signal was concentration dependent only at lower concentrations of HT61. No increase in fluorescent release was observed when HT61 reached concentrations higher than 20 µg/ml.

**Figure 5:** HT61-induced cytoplasmic membrane permeabilization determined by the DiSC3(5) assay. Non-multiplying and log phase MSSA were incubated with DiSC3(5) to a final concentration of 0.4 mM until no more quenching was detected, which was followed by addition of 0.1 M KCl. Different concentrations of HT61 were incubated with non-multiplying MSSA (A) and log phase MSSA (B). The changes in fluorescence were monitored at various time points. The data was confirmed in two independent experiments.

We then examined the ultra-structure of *S. aureus* by transmission electronic microscopy after treatment with the drug. As shown in Fig. 6B, after addition of HT61 for 10 minutes, the cell membrane was disrupted and the cytoplasm leached out into the extracellular space. In addition, we noticed that, after treatment of HT61 at higher concentration, the cell wall was nicked (Fig. 6C and Fig. 6D) and the cell contents were expelled.

**Figure 6:** Thin sectioned electron micrographs of *S. aurues* analyzed by transmission electron microscopy. The cells were fixed 10 minutes after HT61 treatment. A. normal *S. aureus* cells. B. HT61 at 10 µg/ml. C. HT61 at 20 µg/ml. D. HT61 at 40 µg/ml. The scale bar is 0.2 µm.

### HT61 kills non-multiplying MSSA and MRSA on mouse skin

In an attempt to develop HT61 as a topical agent to clear MSSA and MRSA, we investigated if HT61 killed MSSA and MRSA on mouse skin. Two mouse skin models were used. The first model was the superficial skin bacterial colonisation model. Log phase or stationary phase MSSA or MRSA were applied onto the intact skin of live mice at 10^7^ CFU per 2 cm^2^ followed by immediate treatment with 45 µl of HY50A (gel containing 1% HT61) or 45 µl of Bactroban ointment (GlaxoSmithKline containing 2% mupirocin) or 45 µl of placebo. As shown in Fig. 7, after two hours of treatment, HT61 removed 100% stationary phase MSSA (Fig. 7A) and 93% stationary phase MRSA (Fig. 7B) on the mouse skin. In contrast, Bactroban showed no activity against the same bacteria (Fig. 7A and 7B). When log phase MSSA was applied on to mouse skin, Bactroban was more effective than HT61 showing 100% reduction of the bacteria, whilst HT61 killed 55% of the bacteria on the skin (Fig. 7C).

**Figure 7:** Effect of HT61 against MSSA and MRSA in a murine skin bacterial colonization model. Stationary phase MSSA (A) and MRSA (B) were applied onto 2 cm^2^ skin area followed by addition of HT61 gel, Bactroban and placebo (control) for 2 hours. Log phase MSSA were treated with HT61 gel, Bactroban and placebo (control) for 2 hours on mouse skin (C). The data has been repeated twice.

The second model which was used is the mouse superficial skin bacterial infection model [19] in which a bacterial infection is initiated with 10^7^ log phase MSSA or MRSA after removal of the upper epidermal layers. As shown in Fig. 8A, no increased growth was seen after infection, the bacterial numbers on the infected skin were constant during the first 24 hours, then gradually decreased. Treatment with HT61 and Bactroban was initiated after 24 hours of infection during which the bacteria remained stationary phase. As shown in Fig. 7, HT61 reduced 2.91 logs of MSSA (Fig. 8B) and 1.87 log of MRSA (Fig. 8C) after treatment for 24 hours. In contrast, mupirocin reduced 0.86 logs of MSSA and 0.13 logs of MRSA respectively.

**Figure 8:** Effect of HT61 against MSSA and MRSA in a murine skin bacterial infection model. A. After tape-stripping the skin, log phase MSSA was applied onto the skin area. At different time points CFU counts of the bacteria were determined. The arrow indicates the point which the treatment was initiated. B. Treatment of HT61, Bactroban and placebo (control) against MSSA and C. Treatment of HT61, Bactroban and placebo (control) against MRSA. **, P<0.01. The data has been repeated twice.

### Toxicity of HT61

Minipig skin was used to test HT61 for potential dermal toxicity. These studies were conducted by LAB Research (Scantox Denmark). After 14 days of administration of HT61 (1% gel formulation) to 10% of the body surface of each animal, no treatment related adverse events were seen in clinical observations such as irritation, inflammation, itching and sensitization, body weight and food consumption (data not shown). Furthermore, no changes were seen before termination of treatment in clinical chemistry, haematology, urinalysis and during ophthalmoscopy or during electrocardiographic examination, at necropsy or at histopathological examination. No changes were seen at histopathological examination of the skin. Toxicokinetic evaluation verified that the animals had been treated with HT61. An accumulation of HT61 was seen between day 1 to 14 and this may be due to saturation of the skin. Based on the Cmax and AUC0-24h values, no dose proportionality was observed. No consistent gender related differences were seen, although the values for the female animals seemed higher.

## Discussion

Changing the target of drug development from multiplying to non-multiplying bacteria creates a new set of opportunities for antibiotic development. In particular, novel classes of antibiotics can be discovered which show bactericidal activities against non-multiplying bacteria, but may be less potent against multiplying bacteria. HT61 is the first example of the selection of an antibiotic from the beginning of the development process which is active against non-multiplying bacteria. Interestingly, HT61's activity against multiplying bacteria is not as potent as current marketed antibiotics, and so it would have been rejected by conventional anti-multiplying screening tests. In our experience, this is not an isolated example, and we anticipate that this new method will produce many new classes of antibiotics.

HT61 is a narrow-spectrum antibiotic which is only effective against Gram positive bacteria. HT61 is particularly active against *S. aureus* including 162 strains of MRSA which represent the major pathogens in the world, and those that carry the Panton-Valentine leukocidin gene. HT61 can act on multiplying bacteria, but its MIC is higher than that of the marketed antibiotics. However, it showed significant potency against non-multiplying organisms. For MSSA and MRSA at 10^7^ CFU/ml, the concentration (MSC_50_) used to reduce half of the initial bacterial load was 2.5 µg/ml and the concentration to achieve a 99% kill (MSC_99_) is 4.5–6 µg/ml. The concentration required to achieve a complete kill was 12.5 µg/ml. The potency of HT61 was significantly higher than that which has been reported for the anti-stationary phase agent daptomycin [20] that required 50 µg/ml to completely kill stationary phase MSSA and MRSA (Fig. 2). Due to its combined action against multiplying and non-multiplying bacteria, HT61 has the potential to treat an infection with a mix of organisms that are in different growth phases. Although HT61 has lower bactericidal activity against multiplying bacteria than marketed antibiotics, it is used in such a high concentration in its topical formulation (currently 1% v/v, 10 mg/ml) that this should compensate for this weakness.

The precise mode of action of HT61 has not been demonstrated as yet. However, cell membrane depolarization of *S. aureus* was observed after treatment with HT61. The compound acts on the bacterial cell cytoplasmic membrane by disruption of *S. aureus*'s cell membrane potential, and this leads to the release of the cellular contents. Furthermore, HT61 also acts on the bacterial cell wall. After 10 minutes of treatment, the cell wall structure is nicked when HT61 is used at higher concentrations. This suggests that HT61 has several mechanisms of action, whose targets lie in the bacterial cell cytoplasmic membrane and the cell wall. Further investigation into the mode of HT61 action is under way in our laboratory.

The most important property of HT61 is its activity in animal models of *S aureus* skin infection. In animals infected with multiplying and non-multiplying bacteria which had been applied to normal skin, 10^6^ or more bacteria were killed by a single application of the antibiotic at a 1% concentration. In contrast, mupirocin at 2% concentration failed to kill the non-multiplying organisms. In animals which had skin partially stripped prior to application of bacteria, the bacterial load remains relatively constant after infection during the first 48 hours, indicating that the bacteria stay non-multiplying or slowly multiplying. A 10^2^–10^3^ CFU bactericidal effect was also seen with HT61 but Mupirocin barely had any effect.

Examination of the clinical usefulness of HT61 in man is now under way. This antibiotic will be used topically at high concentration (10 mg/ml). At these concentrations, it is anticipated that it will be bactericidal for both multiplying and non-multiplying bacteria. This means that it may be useful as a stand-alone antibiotic. On the other hand, better results may be obtained by using it in combination with another antibiotic which is active against multiplying bacteria. The combination should remove the entire population of targeted bacteria. The best examples of combinations of anti-multiplying and anti-non-multiplying antibiotics are in tuberculosis chemotherapy [21], [22], [23], [24], where isoniazid (kills multiplying bacteria) and pyrazinamide (kills non-multiplying or persistent organisms), are used side by side, together with other antibiotics such as rifampicin and ethambutol.

HT61 will be used clinically to decolonize the nose for *S aureus*, including MRSA. Potential advantages over the market leader, mupirocin, are as follows: Firstly, HT61 is active against mupirocin resistant bacteria. In countries such as Spain, mupirocin resistance is so high, that it is no longer used in many hospitals [25]. It is likely that widespread use of mupirocin in the rest of the world will result in an increase in mupirocin resistance in many countries. Mupirocin resistance can occur at high level or low level [26], [27], [28], [29], [30]. This type of resistance is associated with bacteriological relapse in the nose within a shorter period of time than for sensitive strains [31]. Whilst low level mupirocin resistance can be induced in vitro in the presence of increasing concentrations of mupirocin [32], [33], we have demonstrated that no HT61 resistant strains were obtained after 50 passages of selection during the period of log phase and stationary phase growth. Secondly, HT61 may be able to shorten the duration of therapy in situations where non-multiplying bacteria are present. In comparison to marketed antibiotics, HT61 is about one million times more potent against non-multiplying *S. aureus*. In vitro and in animal models, HT61 shortens the duration of therapy, but it is not known whether this will occur in humans. However, it is likely that populations of bacteria, other than multiplying ones in log phase exist on the human skin. For example, if all the bacteria on the human skin were multiplying, it would be expected that overnight growth would be so rapid that colonies would be visible in the morning. Clearly this is not the case, which suggests that, perhaps due to lack of nutrients and other essential growth factors, bacteria do not usually multiply rapidly on human skin, or in the nose. Indeed, we show (Fig 8A) here that bacteria on mouse skin after infection did not sustain growth. In other diseases, such as tuberculosis [34], bacterial endocarditis [35], [36], [37] and biofilms on intravenous catheters [38], [39] mixed populations of bacteria are known to co-exist. Whether this also applies to the skin and to the nose is not known. Thirdly, it may be possible to reduce the rate of emergence of resistance. Shortening of the course of antibiotic therapy itself may reduce the emergence of resistance because it is known that long courses can be associated with the emergence of resistance, for example due to poor patient compliance. HT61 acts fast, and this may reduce the chance of emergence of resistance. This antibiotic also acts against the cell membrane and the cell wall, and resistance emergence to this compound may be lower than other antibiotics which target a single enzyme, such as rifampicin or mupirocin [40], [41], [42], [43], [44]. Combination of HT61, or similar compounds with antibiotics which kill multiplying bacteria, may prolong the useful life of such partner antibiotics because, if the combination of the two antibiotics kill the entire bacterial target population faster than each on its own, the rate of resistance emergence may be slowed [45], [46]. After all, dead bacteria cannot mutate. Another way of prolonging the useful life of existing antibiotics, such as mupirocin, would be to use the existing antibiotic once only in an individual, and then use HT61 for treatment of relapses. In this way, repeated exposure of bacteria in one individual, a sure way to induce resistance, would be limited. Fourthly, HT61 may lengthen the period before relapse occurs. In the nose, *S. aureus* including MRSA can be removed by the use of mupirocin [31]. However, if the bacteria are resistant to mupirocin, relapse occurs within a few weeks [47]. For sensitive organisms, there is a 30% relapse rate at three months, and by six months, 50% have relapsed [48]. The fact that patients who are colonized with mupirocin resistant bacteria relapse early with mupirocin resistant strains suggests that these persist in the nose. It is not known what proportion of patients who relapse with sensitive bacteria, do so as a result of relapse of persistent bacteria in the nose, or auto-infection from another site in the body, such as the finger. Since the initial strains are usually the same as the relapse strains [49], it is thought re-infection from other people or other sources is less likely than autoinfection.

In conclusion, this paper describes the properties of a novel antibiotic which has been produced by a new approach, namely, by selecting, from the beginning of the discovery process, compounds which are active against non-multiplying bacteria. This method should be able to yield many new classes of antibiotic. In addition, these antibiotics may be able to reduce the rate of emergence of resistance, shorten the duration of therapy, and reduce relapse rates.

## Materials and Methods

### Bacterial strains and growth conditions

Bacterial strains used in this study are list as following; Oxford, *S. aureus* NCTC 6571 (methicillin-sensitive), methicillin-resistant *S. aureus* (MRSA NCTC 12493), MRSA strains (clinical isolates from St George's Hospital, London), *S. epidermidis* (NCTC 5955), *S. pyogenes* (NCTC 10867), *S. agalactiae* (NCTC 8542), *P. acnes* (NCTC 737) and Gram-negative bacteria, such as *E. coli*, *K. aerogenes* and *P. aeruginosa* (clinical isolates from St George's Hospital, London). The strains of *Staphylococci* and Gram-negative bacteria were grown in nutrient broth (Oxoid) or on blood agar plates and the strains of *Streptococci* and *P. acnes* were grown in brain heart broth (Oxoid) or on blood agar plates.

### Antibiotics and drug-like compounds

Antibiotics were used as follow: Augmentin (1.2 g containing co-amoxiclav 1000/200, GlaxoSmithKline), Azithromycin (Zithromax™ suspension, 40 mg/ml, Pfizer), Levofloxacin (Tavanic® 5 mg/ml Hoechst Marion Roussel), Linezolid (2 mg/ml Zyvox, Pharmacia), daptomycin (Cubicin, Novartis) and Mupirocin (Sigma). 56 quinolone-like compounds were obtained from Bionet Research, Butt Park Ltd, Maybridge, Enamine and Specs. HT61 was synthesed by Argenta Discovery UK. Stock solutions of the tested compounds were prepared in dimethyl sulfoxide to 10 mg/ml.

### Susceptibility test of antibiotics against exponentially growing bacteria

The minimum inhibitory concentration (MIC) was determined by the broth dilution method in Iso-Sensitest broth (Oxoid) following the Clinical and Laboratory Standards Institute guidelines for broth microdilution MIC. A physiological level of 50 mg/L Ca^2+^ was supplemented to Iso-Sensitest broth when testing daptomycin. MIC value was defined as the lowest concentration resulting in 90% inhibition of growth.

### Susceptibility test of antibiotics against stationary phase non-multiplying bacteria

The methicillin-sensitive *S. aureus* (MSSA), methicillin-resistant *S. aureus* (MRSA), *S. epidermidis* and Gram negative strains were cultured in nutrient broth over-night at 37°C. Two hundred microliters of the overnight cultures were used to inoculate 100 ml of nutrient broth. Then the cultures were continuously shaken at 110 rpm at 37°C for 10 days. For growth of *S. pyogenes* and *S. agalactiae*, a serial of 10 ml brain heart broth was inoculated with the overnight cultures, and then the cultures were incubated without shaking for 6 days. For growth of *P. acnes*, the broth cultures and the blood agar plates were incubated under anaerobic conditions for 5 days. Viability was determined by plating 100 µl of serial dilutions onto nutrient agar (Oxoid) plates or blood agar plates and was expressed as colony forming units (CFU) per milliliter. The CFU was counted using aCOLyte colony counter (Synbiosis) and analyzed using the software came with the counter. To test antibiotic activities against stationary phase non-multiplying bacteria, the 5–6 day old cultures were washed with phosphate buffered saline (PBS) and diluted in the same buffer to 10^6^ or 10^7^ CFU/ml which was served as cell suspension for drug sensitivity test. For testing of daptomycin, a physiological level of 50 mg/L Ca^2+^ was supplemented. The cell suspension was added in each well of a 96-well microtiter plate incubated with different concentrations of the drugs in triplicate to a final volume of 300 µl. At different time points after drug incubation, the cultures were washed three times with PBS and were resuspended in the original volume. The activities of the drugs against stationary phase non-multiplying bacteria were determined as minimum stationary phase-cidal concentration 50 (MSC_50_) [5] which is defined as the concentration of the drug leading to a reduction in half of the initial bacterial counts and minimum stationary phase-cidal concentration 99 (MSC_99_) which is defined as the concentration resulted in reduction of 99% initial bacterial counts.

### Multistep selection of resistance

The bacteria were cultured in nutrient broth over-night at 37°C. 20 microlitres of the overnight culture were used to inoculate 10 ml of nutrient broth which was incubated for 5–6 days. The drug was added into the stationary phase culture to a concentration which was 2-fold below its MSC_50_. After two days of exposure, 200 µl of the culture was added to 10 ml of fresh nutrient broth, at the same time the drug was added to the final concentration which was 2-fold below its MIC. After drug exposure for 4 days, single colonies were picked and sensitivity test was carried out against both stationary phase non-multiplying and log phase cultures. During this procedure, the drug was exposed to both log phase and stationary phase cultures. Fifty passages of drug exposure, as described above, were performed to select drug resistant bacterial strains.

### Fluorescent assay to measure cytoplasmic membrane potential

Cell membrane permeability was measured using a fluorescent assay as described previously [50]. Log phase or stationary phase cultures were harvested and washed with PBS. The bacterial cells were resuspended with PBS to an optical density of 0.05 at 600 nm. The cell suspension was incubated with 0.4 µM DiSC3(5) (Dipropylthiacarbocyanine) (Sigma), a membrane potential sensitive cyanine dye, until a stable (approximately 90%) reduction in fluorescence was reached as a result of DiSC3(5) uptake and quenching in the cell due to an intact membrane potential. Then 100 mM KCl was added into the cell suspension to equilibrate the intracellular and external K^+^ concentrations. The samples were placed into wells of a 96 well flat bottom fluorescence microtitre plate (Fischer Scientific UK) followed by addition of different concentrations of drug in triplicates. Fluorescence was monitored using a fluorescence spectrophotometer (Applied Biosystem) at an excitation wavelength of 622 nm and an emission wavelength of 670 nm. The induction of fluorescence, which resulted from the disruption of the cytoplasmic membrane by different concentrations of drugs, was recorded. The background was subtracted using a control which contained only the cells and the dye.

### Electron Microscopy

Bacterial cultures were harvested and fixed with a fixation solution containing 2% formaldehyde and 2% glutaraldehyde, 0.2 M sucrose in 0.1 M cacodylate (pH 6.9) buffer. Sample processing, sectioning and examination of the transmission electron microscope were performed in the Ultrastructural Imaging Unit, King's College London.

### Superficial skin bacterial colonization and infection models

The skin bacterial colonization and infection models were performed using female ICR mice (6 to 8 weeks old) obtained from Harlan, UK Ltd. The animal husbandry and animal care guidelines were followed according to the Animals Scientific Procedures Act, 1986 (an Act of the Parliament of the United Kingdom 1986 c. 14). The study was specifically approved by the animal ethical committee of St George's University of London. For the intact skin bacterial colonization model, ICR mice were anesthetized by intraperitoneal injection of 200 µl of a 1∶1∶2 mixture of 100 mg/ml ketamine hydrochloride, 20 mg/ml xylazine, and sterile water. The fur of the mice on the back was removed by an electric clipper. A two cm^2^ skin area was marked with a marker pen and log-phase or stationary phase cultures (20 to 30 µl) were added on the 2 cm^2^ area. The bacterial suspension on the skin was allowed to dry for 20 minutes. Treatment of the bacteria was performed by spreading 45 µl of gels or ointment on the skin. The superficial damaged skin infection model was performed as described previously [19] with the following modifications. After anesthetizing the mouse and removing its fur on the back, an area of 2 cm^2^ skin is tape stripped using an autoclave tape. The skin was striped 10 times in succession. This procedure damaged the skin by removing the top dermal layers, which became red and shiny, but without observable bleeding. Buprenorphine was given at 0.2 mg/kg body weight during the anesthetic period and every 12 hours for up to 3 days to reduce pain. Bacterial infection was induced by the addition of 10 to 25 µl of log phase culture containing 10^7^ bacterial cells on the stripped skin. At 24 hours after infection, treatment with gels or ointment was initiated. At different time points after infection and treatment, 3 or 4 mice were sacrificed by cervical dislocation. The skin, approximately 2 cm^2^ was cut and added to 2 ml tubes which contained 1 ml water and glass beads (1 mm). The skin was homogenised using a reciprocal shaker (Fisher Scientific UK) for 45 second (6.5 speed). Antibiotic remaining on the skin was removed by washing 3 times with water. CFU counts were performed on serial dilutions of the homogenates.

### Dermal toxicity study

The dermal toxicity of the compounds was performed by LAB Research (Scantox Denmark). Twenty-four Göttingen SPF minipigs (12 males and 12 females) were used for the study which were obtained from Ellegaard Göttingen Minipigs ApS, Denmark. The animals were approximately 3 months old and the body weight was 6.0 to 8.4 kg. They were allocated to 4 groups each consisting of 3 males and 3 females. HT61 was administered daily by dermal application to for 14 days. The dose for the treatment was 1 g/kg/day on 10% of the body surface area. Clinical signs, dermal reactions and food consumption were recorded daily. The body weight was recorded weekly, and in addition, on the day of necropsy.

Before and after treatment, blood and urine samples were taken from all animals for clinical chemistry, haematology and urinalysis. Also the animals were subjected to an electrocardiographic and ophthalmoscopic examination. Blood taken from day 1 and day 14 was also used for toxicokinetic analysis. At the end of the experiment, the animals were anaesthetised, euthanized by exsanguination and subjected to macroscopic necropsy. Selected organs or tissues were weighed, sampled, fixed and examined microscopically.
